# Dynamic Mechanism and Decision Analysis of Urban Exhibition Tourism Development Based on High-Performance Computing

**DOI:** 10.1155/2022/3806752

**Published:** 2022-04-06

**Authors:** Hongzhen Wan

**Affiliations:** School of Management, Guangdong Industry Polytechnic, Guangzhou 510300, China

## Abstract

MICE tourism has received the attention and support from relevant departments and tourism industry with the growth rate of recent years. In this paper, the dynamics mechanism of urban exhibition tourism development is studied by using high-performance computing, and the dynamics mechanism model of exhibition tourism is constructed. To improve the performance, the solution constructed in the adaptive joint algorithm is used as the initial solution, and then the initial solution is improved using the method proposed by the new neighborhood strategy. It promotes the development of MICE tourism and urban MICE tourism by combining research on theoretical aspects related to tourism development, such as the relationship between tourism development and exhibition, and the development dynamics and stages of MICE tourism. The research results show that, in the assessment of the development mechanism of urban MICE tourism, tourism resources, economic, and policy factors have a relatively large weight, among which the weight coefficient of tourism resources factor is 0.2411. It can be seen that the development power of MICE tourism should start from tourism resources, so that the development power mechanism of urban MICE tourism can be optimized and improved, which not only provides new methods and new ideas for the transformation and upgrading of tourism industry but also promotes tourism enterprises and related departments to creatively develop tourism resources and design competitive tourism products, so as to improve the supply quality of MICE tourism, and then continuously promote the process of supply-side reform of MICE tourism.

## 1. Introduction

Scheduling and scheduling tools for high-performance computing (HPC) machines have a key role in mapping jobs to available resources, trying to maximize performance and quality of service (QoS). Bridi et al. demonstrated the first search-based HPC machine job allocation and scheduling method, working in a production environment. The scheduler is based on constraint programming, which is an effective programming technique for optimization problems. Tests on various operating conditions show that, in midlevel HPC machines equipped with the most advanced business rules-based scheduler, waiting and QoS have been significantly improved. In addition, Bridi et al. analyzed the conditions under which their method was superior to commercial methods to create a combination of scheduling algorithms that ensure robustness, flexibility, and scalability. Although their method has certain reference value for the study of this article, it is of little value [1]. Computational models can easily promote the mechanical understanding of multiscale biological processes, such as cell proliferation in constantly changing biological tissues. Although there are tools for constructing and simulating multiscale models, the statistical inference of unknown model parameters is still an open question. Jagiella et al. demonstrated and benchmarked the Parallel Approximate Bayesian Computing Sequential Monte Carlo (pABC SMC) algorithm, which is tailored for high-performance computing clusters. Their research proved the principle of robust data-driven modeling of multiscale biological systems, and the feasibility of multiscale model parameterization through statistical inference. The algorithm is too complicated, and errors may occur in the calculation [2]. Wang et al. discussed the design trade-offs of extremely scalable system software. They proposed a general system software classification method by deconstructing general HPC system software into its basic components. They provided a system method for building scalable system software by decomposing it into basic components, allowing system software to be classified according to the characteristics of these components for design evaluation through simulation or actual implementation. The results show that it helps to lay the foundation for the development of next-generation HPC system software for extreme scale. But this research is still in its infancy, and it is too basic [3]. The high-performance computing (HPC) community has spent decades developing tools and teaching practitioners to use the power of parallel and distributed computing. In order to create a scalable and flexible educational experience for practitioners at all stages of their careers, Mullen turned to Massive Open Online Courses (MOOC). He introduced in detail the design of a unique self-paced online course, and the course materials are presented through the lens of common HPC use cases and parallelization strategies. Using a personalized path, he teaches researchers how to identify the consistency between scientific applications and traditional HPC use cases so that they can focus on learning parallelization strategies that are critical to their workplace success. However, the high-performance computing method he proposed is not specific enough to be discussed in depth [4]. Fu's et al. research examines the potential dimensions of place attachment in the exhibition environment and its impact on participant satisfaction. The study took the China (Shenzhen) International Cultural Industry Expo as a case and proposed and tested a series of multiple intermediary models, divided into two groups: first-time participants and repeat participants. The exhibition attachment determines a function-emotion-identity sequence, examining direct and mediating effects and multiple group comparisons. Although most hypotheses have been confirmed, emotional attachment plays a negative role in predicting exhibition satisfaction, and visit frequency shows significant differences in the impact of exhibition dependence on satisfaction. The research provides specific theoretical and management enlightenment for the exhibition attachment and exhibition satisfaction of the participants. However, the model they put forward is too dependent on the subjective opinions of users and cannot objectively obtain the satisfaction of participants [5]. Lai and Wong developed a ternary reciprocal causality model to study how the knowledge created by customers affects the quality of the relationship and guarantees the perceptual performance of the report. Partial least squares analysis was performed on the data collected by 395 exhibitors in Macau. The results show that the participation of exhibitors in the preparation work has a positive impact on the three factors of relationship quality (satisfaction, trust, and commitment), and these three factors have a positive impact on the perceived performance of the report. Compared with exhibitors at public exhibitions, trust has a greater impact on exhibitors' commitments at trade shows. Research shows the integration of relationship quality theory, customer engagement theory, and social knowledge theory. Only for the three factors of the quality of exhibition participation relations, further research can be done. Yi's research draws on the theory of place attachment and puts forward an innovative concept of exhibition attachment. Based on an in-depth literature review, a conceptual model of exhibition attachment was constructed, including push/pull motivation, attachment, and loyalty. To test the model, empirical data was collected from the participants of the trade show. The results show that there is a certain degree of correlation between the participants' push motivation and pulling motivation. Pulling motivation has a significant impact on exhibition dependence, which in turn has a positive and strong impact on the identity of the exhibition. The push-pull motives he studied have little correlation [6]. Harris and Dieringer conducted an economic analysis of a proposed zoning change that would allow the City of Treasure Island, Florida, to attract more visitors. The proposed zoning change will result in hotel renovations and new hotel construction in Treasure Island, Florida. Harris uses tax analysis to understand how this change will increase taxable property values as well as increase tourism development tax revenues [7]. Giampiccoli et al. explored the intersection between sustainable tourism and community-based tourism (CBT) and revealed a serious mismatch in the concept of sustainability and that addressing its negative environmental impacts is a fundamental requirement for tourism. A. Giampiccoli argues that sustainability in tourism should be an intrinsic and universal principle that governments should implement for all forms of tourism. In fact, traditional tourism causes most of the environmental damage and because of this, it should upgrade its role to become a solid promoter of sustainable measures that promote environmentally friendly and sustainability-friendly practices [8]. Wang et al. proposed a method to supplement fixed lockers with mobile parcel lockers to meet last-mile delivery needs. With the objective of minimizing operational costs, the location and route optimization problems of mobile delivery lockers are integrated into a nonlinear integer programming model. Embedded GA has been developed to simultaneously and optimally determine the location of delivery points, the number of mobile parcel lockers required at each delivery point, and the schedule and route of mobile parcel lockers [9]. Li et al. proposed a novel combined parametric modeling and design optimization technique for microwave components using neural networks. The proposed technique provides an iterative mechanism between artificial neural network model training and design optimization updates. This iterative mechanism is fully automated and does not require human intervention. In addition, the proposed technique overcomes the limitation of common artificial neural network optimization strategies, where the fixed training area of the artificial neural network model limits the degrees of freedom for design optimization. The proposed technique automatically expands the ANN training region until an optimized solution satisfies the user design specification [10]. In order to improve the thermal efficiency of blast furnace to achieve the goal of energy saving and consumption reduction, Zha Ng and Li optimized the blast furnace combustion control process by collecting a large amount of field data and introducing isolated point removal strategy for preprocessing with semisupervised clustering algorithm. The method has been experimentally validated and shows significant energy savings compared with the traditional data preprocessing strategy [11]. Wang et al. proposed a multiobjective evolutionary algorithm based on a decomposition-based differential evolutionary strategy to solve the multiobjective model. A series of nondominated solutions are obtained, which represent the optimal spare parts supply solutions. In order to measure the performance of these solutions comprehensively, suitable quantitative metrics are selected and the efficiency of the obtained optimal solutions is evaluated using a cross-efficiency data envelopment analysis (DEA) model based on secondary objectives [12]. Ramazan proposed an adaptive particle filter (APF). In the APF, the adaptive fuzzy square root untraced Kalman filter (AFSRUKF) is used to generate the proposed distribution. In APF, the resampling process is done based on particle swarm optimization (PSO) in order to increase the diversity of particles. With this resampling strategy, particles with small weights are modified to particles with large weights without duplicating and eliminating particles [13].

The innovation of this paper is to use high-performance computing technology to study the dynamic mechanism of urban exhibition tourism development and establish the dynamic mechanism model of urban exhibition tourism based on the theory of tourism dynamic mechanism and tourism stakeholder theory. At the same time, it combines theoretical research and actual cases of city exhibition tourism to analyze and propose implementation plans. According to the evaluation system and the dynamic mechanism of exhibition tourism development, the dynamic characteristics of various types of power are sorted out, the development path is planned, and development suggestions are put forward. According to the weight difference of each factor of the index, the corresponding countermeasures are proposed to provide preliminary theoretical reference for tourism development researchers. From the load balancing scheduling mechanism, the overall load balancing algorithm can be divided into three categories: static load balancing algorithm, dynamic load balancing algorithm, and adaptive load balancing algorithm.

Convention and exhibition tourism is an important direction of world tourism development, an important part of urban tourism, and a model for the development of urban related industries. Convention and exhibition tourism has now become an important channel for economic and trade exchanges between countries. The convention and exhibition industry, including convention and exhibition industry, exhibition industry, and incentive tourism industry, is a huge industry in the world. Related industries with about 1% of the world's total GDP benefit from the report, and the exhibition industry contributes 8% to the global economy. Therefore, the tourism departments of various countries attach great importance to the development of exhibition tourism.

## 2. Optimization of Urban Exhibition Tourism Development

The characteristics of exhibition tourism are that exhibitors have strong spending power, the tourism industry benefits more, tourists stay for a long time, there are more travel opportunities, and there are more potential participants, which can provide a broad platform for the development of the tourism industry.

The developmental dynamic mechanism refers to the organic collection with specific functions formed by the interaction of elements. The internal mode of interaction between elements is the structure of the system, in which each element is organized into a process for a specific purpose. The current research on the dynamic system of tourism development mainly involves the research on the dynamic mechanism of urban tourism development. These studies determine the supply of urban tourism products and the core competitiveness of urban tourism. We will jointly guide the emergence and development of urban exhibition tourism under the interaction of various dynamics such as stimulating the demand for exhibition tourism, protecting the urban environment, and supporting the country.  Figure 1 is a model of the dynamic mechanism of urban exhibition tourism development.

The development of urban convention and exhibition tourism is driven by different forces, so as to realize the rapid development of convention and exhibition tourism. The factors that affect the development of urban exhibition tourism are divided into two types: driving factors (resources, economy, location, services, etc.) and supporting elements (policy, technology, culture, etc.), and their effects on urban exhibition tourism are presented as driving forces and guiding force. The figure shows the law of behavior among various factors affecting the development of exhibition tourism from the analysis of the entire city system. Among them, policy, technology, culture, economy, resources, location, and service are regarded as development driving factors.

The shift-share analysis method usually takes the economic development status of the region where the city is located as a reference, uses the gross national product as an index to evaluate the economic aggregate, and studies the change process of the regional economic industrial structure through the dynamic development process [14, 15]. When constructing the shift-share model, three indicators of the total economic volume of the case are generally selected: the first is the amount of change in the standardization industry department of the case study area based on the average growth rate of the region, that is, the deviation share W; the second is the impact of the structural difference between the case area and the regional economy, that is, the deviation of the industrial structure from the share *R*; the third is the difference in the level of economic activity caused by the difference in economic growth between the various industrial sectors within the region and the corresponding industrial sector in the case, that is, the deviation of competitiveness from the share *L*. Suppose that, in time *s*, in region *A*, the overall economic aggregate and industrial structure of the region have undergone some changes, and suppose that the overall economic aggregate and industrial structure of the region have undergone some changes. Assuming that the economic aggregate of this time period is *T*_all_ and the economic aggregate of the last year is *F*_all_, then the relevant mathematical model of the deviation-share analysis method of area *A* can be expressed as

(1) $$\begin{array}{c} H_{a}=W_{a}+R_{a}+L_{a}=T_{\text{all}}+F_{\text{all}},\\ W_{a}=\frac{T_{a}}{F_{a}}*T_{\text{all}}-F_{\text{all}},\\ R_{a}=\overset{N}{\underset{a=1}{\sum }}\frac{T_{a}}{F_{a}}\times T_{\text{all}},\\ L_{a}=T_{j,a}-\overset{n}{\underset{a=1}{\sum }}\frac{T_{a}}{F_{a}}\times \left(T_{\text{all}}+F_{\text{all}}\right). \end{array}$$

Among them, *W*_*a*_ is the deviation share of region *a*, *R*_*a*_ is the deviation share of the industrial structure of region *a*, and *R*_*a*_ is the competitiveness share of region *a*.

(2) $$\begin{array}{c} {\left(R+L\right)}_{a}=R_{a}+L_{a}=T_{all}-\frac{T_{a}}{F_{a}},\\ \eta =\frac{T_{i,a}}{\overset{n}{\underset{a=1}{\sum }}\times \left(T_{a}/F_{a}\right)\times F_{j,a}}. \end{array}$$

*η* is the regional competition effect index, which can more accurately analyze the status quo of the industrial structure of the economic development of region *a*.

High-performance computing refers to a device with a very powerful computing capability to complete a specified amount of computing work in a short period of time, mainly used to deal with complex calculation problems, and the development dynamic mechanism of exhibition tourism in this paper needs to calculate various dynamic factors in exhibition tourism. At present, high-performance computing is widely used in scientific research fields, such as national defense and military industry, molecular chemistry, computer engineering assistance, global long-term meteorology, weather and disaster forecasting, process improvement and environmental protection, biological information technology, and medical and new drug research. Currently, the data is growing massively, from the Internet of Things to cloud computing, from big data to artificial intelligence, from Bitcoin to blockchain [16, 17], and the information revolution is rapidly promoting the development of the industry, subverting traditional concepts, and affecting around the world. Often companies need to make faster development and greater innovation in their business, accompanied by fast, stable, strong, and more demand for new computing capabilities. In the field of artificial intelligence, the rapid development of deep learning technology represented by graphics, images, audio, and video requires high-performance computing power to provide support [18, 19].

Figure 2 is the general architecture of the high-performance computing hardware platform.

With the deepening of scientific research, fierce competition, and rapid growth of data volume, digital and analog calculations are becoming more and more accurate, and the demand for computer resources is also increasing. Higher and more comprehensive requirements are put forward for data storage, computing speed, response time, and network bandwidth. Simulation has become an indispensable tool for researchers to explore the system without resorting to actual experiments. In any case, increasing the size and accuracy of the model will increase the amount of calculation [20, 21]. Consider computing, storage, and networking from three perspectives. IT mainly includes computer nodes, acceleration nodes, auxiliary nodes, connection nodes, and management nodes. There are three network levels in the network: high-speed computer network, storage network, and management network; separate the management levels inside and outside the area, and the management network system and business system do not share the same level [22, 23]. When the business system fails, the administrator can also manage the server through the offline management network console [24].

From computers, minicomputers, to mainframes, the rapid development of computers is still unable to meet the needs of computing. Scientific computing, network computing, terminal computing, cloud computing, supercomputing, intelligent computing, GPU (Graphics Processing Unit) computing, and other computing modes, concepts, technologies, and applications dominate the progress and development of science and technology. Quantum computing, brain-like computing, borderless computing, human-machine-object ternary fusion computing, data-intensive computing, etc. have brought computing into the multielement era [25, 26]. Calculations allow humans to explore the unknown. The future development is no longer simply a certain technology or a certain type of calculation; it must be a combination of multiple calculations, and multiple theories cooperate with each other to develop together [27].  Figure 3 shows the workflow of high-performance computing.

The terminal allocates the work and sends a message to each node to let them perform their own part of the work. The work is put into the high-performance computing unit and sent to each node at the same time, and each node is usually expected to give a result at the same time as a response. The results from each node are returned to the host application through another message provided by MPI, and then all messages are received by the application.

### 2.1. Balanced Load

Load balancing refers to the processing of a large amount of data requests or a large amount of data requests in a short period of time through resource scheduling and task allocation. It balances the distribution of load and avoids overload, so as to maximize the use of system resources, maximize system throughput, and minimize task idle time. Generally speaking, load balancing is a global optimization scheduling problem. Load balancing scheduling is classified according to types and can be divided into local and global scheduling strategies. Global scheduling strategy is divided into dynamic load balancing and static load balancing; dynamic load balancing is divided into centralized and distributed scheduling strategies, etc. Here from the load balancing scheduling mechanism, the overall load balancing algorithm can be divided into three categories: static load balancing algorithm, dynamic load balancing algorithm, and adaptive load balancing algorithm. The balanced load model is shown in Figure 4.

Supposing a represents an effective task scheduling strategy, then *K*(*a*) represents all the time the task set *K* is executed on the server node *R*, and the goal that the task scheduling needs to meet is to require the optimal span. Here, make *K*(*a*) as small as possible.

Let H denote the set of load balancing indicators, and set *H*={*H*_1_, *H*_2_, ..., *H*_*n*_}; then,

(3) $$\begin{array}{c} H_{i}\left(a\right)=\frac{1}{K\left(a\right)}\overset{s}{\underset{i=1}{\sum }}S_{ij}\times T_{ij}, \end{array}$$

where *i* ∈ {1,2, ..., *n*}, and you can get 0 < *H*_*i*_(*a*) ≤ 1, and suppose that the standard deviation *ϕ*(*a*) of the load index is defined as *ϕ*(*a*),

(4) $$\begin{array}{c} \varphi \left(a\right)=\sqrt{\frac{1}{m}{\left(H_{i}\left(a\right)-\frac{1}{m}\overset{m}{\underset{i=1}{\sum }}H_{i}\left(a\right)\right)}^{2}}. \end{array}$$

According to 0 < *H*_*i*_(*a*) ≤ 1, 0 ≤ *ϕ*(*a*) < 0.5 and *γ*(*a*) is the standard deviation of the load index; then *γ*(*a*) is defined as

(5) $$\begin{array}{c} \gamma \left(a\right)=1-\left(2\times \varphi \left(a\right)\right). \end{array}$$

According to 0 ≤ *ϕ*(*a*) < 0.5, 0 < *λ*(*a*) ≤ 1 can be obtained.

According to the mathematical model, the task scheduling algorithm can be described as looking for a task scheduling strategy that makes *K*(*a*) as small as possible and *γ*(*a*) as large as possible, which is the optimal solution.

In order to improve performance, the solution constructed in the adaptive joint algorithm is used as the initial solution *x*, and then the method proposed by the new neighborhood strategy is used to improve *x*. First, determine and select the last scheduled task on all nodes, and the first improvement has been made. This method involves finding all the inactive time intervals of the node and trying to insert the operation of the selected task while respecting the constraints. The optimal time selection parameter represents the processing time of tasks on all nodes. The processing time from the first to the last vertex of the path is expressed as

(6) $$\begin{array}{c} \text{WL}\left(a,b\right)=\left(\underset{i\in e_{ab}}{\sum }W_{a,b}\right)+W_{i}. \end{array}$$

Among them, *W*_*a*,*b*_ is the collection of all the data before the job; calculate the workload of each operation, and according to the total workload, sort the jobs in the order of the highest workload to the lowest workload.

(7) $$\begin{array}{c} \text{WL}\left(a\right)\left\{\begin{array}{c} \arg\left\{\max_{a\in E\left(a\right)}{\left[\delta_{i}^{k}\right]}^{j}\right\},\\ s>s_{0}. \end{array}\right. \end{array}$$

Among them, *s* represents the information between paths, *δ*_*i*_^*k*^ represents the heuristic distance between them, and *E*(*a*) represents a random number uniformly distributed in [0, 1].

(8) $$\begin{array}{c} \delta_{\text{ij}}\left(a+1\right)=\left(1-g\right)\delta_{\text{ij}}\left(a\right)+\nabla \delta_{\text{ij}},\;0<g<1,\\ \Delta \delta_{ij}\left(a\right)=\overset{ij}{\underset{k=1}{\sum }}\delta_{ij}^{k}\left(a\right). \end{array}$$

When all the data in the job distribution process constructs a complete path from the beginning to the last vertex, each data will be marked to provide pheromone for each directional arc.

(9) $$\begin{array}{c} \nabla \delta_{\text{ij}}^{k}\left(a\right)=\left\{\begin{array}{c} \text{WL}\left(a\right),\left(\text{ij},\text{ea}\right)\in \upsilon^{k}\left(a\right),\\ 0,\text{others}. \end{array}\right. \end{array}$$

### 2.2. Task Division

Task division has a significant effect on data-intensive applications, but its ability to execute complex data structures and control flow instructions is not good. When the problem scale is small or the frequency of use is low, different task division methods are used.

Consider the program running time; suppose *s* is the program running time, *s*_cpu_ is the CPU preprocessing time, *s*_copy_ is the data copy time, *s*_gpu_ is the kernel execution time, and *s*_ret_ is the return time of the abnormal data copy function. Then when the exception copy is not used, there are

(10) $$\begin{array}{c} S=S_{\text{cpu}}+S_{\text{copy}}+S_{\text{gpu}}. \end{array}$$

When using asynchronous data copy, there are

(11) $$\begin{array}{c} s=\max\left\{\left(s_{\text{cpu}}+s_{\text{ret}}\right),\left(s_{\text{copy}}+s_{\text{gpu}}\right)\right\}. \end{array}$$

Neglecting the execution time of kernel and the return time of the asynchronous data copy function, it can be expressed as

(12) $$\begin{array}{c} s=\left\{\begin{array}{c} s_{\text{cpu}}+s_{\text{copy}},\\ \max\left\{s_{\text{cpu}},s_{\text{copy}}\right\}. \end{array}\right. \end{array}$$

It is not difficult to see from the formula that when the preprocessing time is close to the data copy time, the use of asynchronous data copy can shorten the program running time by half. The concurrent operation of data copy and execution has the effect of the pipeline, which can effectively hide the delay and improve the report and document classification program performance.

For a single job in the system, without considering the impact of other jobs, there may be a time interval between the occurrence of communication events during its execution. The analysis of communication characteristics in the time dimension of parallel applications mainly focuses on the interval distribution of the communication interval, and the interval is

(13) $$\begin{array}{c} g\left\{f\left(p,w+1\right)\right\}-f\left(p,w\right)=P\left(a\right),\\ W\left(a\right)=\left\{\left(w-1\right)f\left(w-1,a\right)-\text{wf}\left(w,a\right)\right\}, \end{array}$$

where *g* represents the mathematical expectation and *P*(*a*) is the proportional coefficient. If the *a* + 1 interval appears in the middle of the previous a interval, it will increase on the basis; then,

(14) $$\begin{array}{c} g\left\{f\left(1,a+1\right)\right\}-f\left(1,a\right)=\varepsilon -P\left(a\right)f\left(1,a\right)\;\left(0<\varepsilon \left(a+1\right)<1\right). \end{array}$$

It can be seen that there is an intersection of the communication intervals of multiple communication events. When there is no noncommunication interval among them, no communication event occurs.

Using the principles and steps of analytic hierarchy process, construct the quantitative evaluation index system of the urban exhibition tourism development dynamic mechanism to determine the weight of its evaluation factors. The development motivation factor is used as the first-level evaluation index, including policy, technology, culture, economy, resources, location, and service, expressed in *T*_1_–*T*_7_. Then the factors under the first-level indicators are used as the second-level indicators, and the detailed evaluation indicators are shown in Tables 1 and 2.

The secondary indicators of the development momentum of exhibition tourism include economics, policies, resources, services, location, technology, culture, and other content. The level of economic and industrial development reflects the inherent support for the development of urban exhibition tourism. The urban economy has the early advantages of urban construction. Convention and exhibition tourism uses typical industries as growth engines. It is understandable that typical industrial development drives urban development. Especially as a tourist city, the development of tourism affects all aspects of urban construction. Therefore, the level of economic development and the development of typical industries directly affect the development of tourist cities. Among them, the stable and healthy development of the exhibition tourism industry requires a good market order, which requires the government to formulate relevant laws and regulations to regulate various commercial behaviors in the industry. On the basis of improving the current industry standards and regulations, the government has formulated more comprehensive qualification assessment standards, evaluation mechanisms, market competition, market supervision, and related laws, regulations, and preferential policies in the exhibition and tourism industry. It is used to coordinate the interest relationship between all parties and prevent the vicious competition in the market caused by the interests of all parties, so as to create a good market order and realize the healthy and stable development of Guilin convention and exhibition tourism.

According to the quantitative nature of the indicators, construct indicators for the dynamic development mechanism of urban exhibition tourism. The first-level indicators are elements of support and promotion, and the second-level indicators are improvements to the first-level indicators, which can more fully reflect the reporting situation of the city, judging the relative importance of each element at each level, and expressing the judgment in the form of a digital table to create a judgment matrix. The structure of the judgment matrix is shown in Figure 5.

By constructing a judgment matrix, calculating the factor weights layer by layer, and then obtaining the ranking of the importance of the factors that affect the complex problem, the evaluation of the development momentum of urban conventions and exhibitions is mainly based on the weight difference of various factors, and the corresponding development path of the convention and exhibition tourism planning will not have a major impact on development trends and changes due to factors such as time.

From the perspective of tourists' recognition, this study established a city exhibition tourism satisfaction evaluation system through questionnaire surveys and expert interviews. Through the analysis of the development factors of exhibition tourism, the development process of urban exhibition tourism is analyzed. The problems and effective ways to improve the competitiveness of city exhibition tourism are put forward. In this task, we distributed 150 questionnaires to different target groups and collected first-hand raw data through the questionnaires. We selected evaluation indicators through on-site visits and inspections, participation in relevant exhibitions, study and research of relevant departments, and the perceived satisfaction of exhibition exhibitors, tourists, and local residents. We used the data collected from the survey to directly collect the original data.  Figure 6 shows a framework for analyzing and investigating MICE tourism satisfaction.

## 3. Optimization Results of Urban Exhibition Tourism Development

The exhibition tourism industry is a huge driving force for urban development and product brand building. With the increasing frequency of economic and trade cooperation and exchanges in various regions, large-scale exhibitions in various cities have become important promoters of economic and trade cooperation, economic introduction, and products going abroad. Convention and exhibition tourism has gradually developed into an important industry in the economic development of each city. At the same time, according to the increasingly fierce competition in urban development location and the continuous segmentation of products and markets, it has a clear position in the development of exhibition tourism. The positioning of these cities for the development of exhibition tourism undoubtedly determines the trend and positioning of the city in the future development. It also determines the trend pattern of future exhibition tourism development and the overall strength of the city's development. The tourism development of city A in recent years is shown in Figure 7.

Figure 7 shows the tourist arrivals and growth rate of city A in recent years. It can be seen that, from 2015 to 2019, the annual tourist arrivals and tourism growth rate of city A have increased significantly. According to statistics, the annual profit of exhibition tourism in the tourism market of city A is more than 20%–25%, and there are more than 400 large-scale exhibitions each year, which is in the upper reaches of the country.

From Figure 8, combined with the number of tourists in Figure 7, it can be seen that the exhibition tourism market in city A has shown great development potential. Among tourists, conference tourists account for 10.3% of the total tourists, second only to vacation and sightseeing tours. Its unique tourism resources, rich leisure, and entertainment activities and perfect service system have exerted a strong pull on the development of exhibition tourism in city A.

According to the first- and second-level evaluation indicators of the development momentum of exhibition tourism constructed in the previous article, the weight coefficients contained in each indicator are calculated.  Table 3 is the judgment matrix of the first-level index weight coefficient, which determines the weight of each evaluation factor and then improves and optimizes its development motivation mechanism, so that the exhibition tourism can develop in a healthy and orderly manner.

Analyzing the weights of the first-level evaluation indicators, it can be seen that tourism resources and economic factors and policy factors have a relatively high weight. Among them, the weight coefficient of tourism resources is 0.2411, which has the highest weight. After the judgment and analysis of the index matrix, and the consistency test of the single-level and total rankings, the weight coefficients of the secondary indicators are analyzed.  Figure 9 shows the weights of the secondary evaluation indicators of the exhibition tourism development dynamic mechanism.

From the perspective of system science, the analysis of tourism power mainly includes the attraction system based on tourism demand, the attraction system based on tourism supply power, the tourism promotion power system, and the supporting power formed by its development. Therefore, the development of exhibition tourism has common characteristics. Secondly, from the internal analysis of the dynamic system, these factors are not independent, nor are they purely linear. There is a certain causal effect and feedback influence between them. Refer to the previous evaluation index composition, combined with the relevant data of the current situation, to obtain the power index of the power factor index of the exhibition tourism development. The power index and the index assignment are shown in Figures 10 and 11.

Use index assignment to determine the weight of dynamic factors and determine the degree of influence of different dynamic factors on the development of exhibition tourism. That is, the evaluation of the dynamic factor and the index assignment mainly adopt the analytic hierarchy process.

After calculating the weights of the indicators, the indexes of the dynamic factors at various levels are obtained. It can be seen that although the tourism resources of city A are relatively rich, the actual power is more, and the location and environmental factors are relatively strong. However, in view of the current driving force of the development of exhibition tourism in which resources play a major role, the driving force of resource factors on the development of exhibition tourism is still relatively strong.

The most important thing in MICE tourism is the degree of satisfaction of tourists during their travel. Only when the tourists are satisfied can they attract more tourists to travel. Through the survey of tourist satisfaction in exhibition tourism, we can analyze and study the development direction of Hu Zhan tourism and the improvement of exhibition tourism service quality.  Figure 12 is the questionnaire analysis on the satisfaction of exhibition tourism.

In the questionnaire for residents' satisfaction, urban factors, exhibition facilities, exhibition environment, tourism resources, tourism costs, and other indicators are set to analyze the satisfaction of exhibition tourism. Through the analysis of survey statistics, we can use evaluation indicators to make it clearer that customers attach great importance to those issues in the development of exhibition tourism, but the customer perception evaluation is very low. These need to be strengthened and improved by the exhibition management department and related organizers.

## 4. Conclusions

This paper analyzes the dynamic mechanism of urban exhibition tourism development through high-performance computing and conducts research on the optimization countermeasures of exhibition tourism. Under the premise of clarifying the differences in the development of city convention and exhibition tourism, the dynamic factors of the development of convention and exhibition tourism industry are analyzed. Regarding the main characteristics and content of the seven main driving factors of exhibition tourism development, refer to the relevant evaluation index system to subdivide the driving factors of exhibition tourism development, economic factors, selection policy factors and resource factors, and other location factors. Taking into account the factors of the investigation, the concept and composition of each element are refined layer by layer, and finally a multifactor evaluation system for the development of exhibition tourism is formed. We used surveys and detailed layering procedures to determine the weights of all levels of measurement. From the weighted results, we can see the characteristics of the power structure of the city's exhibition tourism in the emergence stage. The load balancing algorithm is mentioned in the article, and load balancing is a global optimization scheduling problem. Combined with the principle of dynamic factors, it analyzes and summarizes the characteristics and main development paths of exhibition tourism under the combined effect of various factors. However, there are still some shortcomings in the article research, such as the lack of depth in the current research on the dynamic mechanism of the development of exhibition tourism in the city, and the selection of evaluation factors and mechanism research on the dynamic mechanism of exhibition tourism are not perfect. We hope it can be improved in the future work.

## Figures and Tables

**Figure 1:** The dynamic mechanism model of city convention and exhibition tourism development.

**Figure 2:** General architecture of high-performance computing hardware platform.

**Figure 3:** High-performance computing job workflow.

**Figure 4:** Balanced load model.

**Figure 5:** Evaluation index judgment matrix.

**Figure 6:** The analysis and research framework of exhibition tourism satisfaction.

**Figure 7:** Number of domestic and foreign tourists in Hangzhou from 2015 to 2019.

**Figure 8:** *x* city's tourist purpose in recent years.

**Figure 9:** The weight of the secondary evaluation index of the development dynamic mechanism of exhibition tourism.

**Figure 10:** Motivation factors and index assignments for the development of exhibition tourism.

**Figure 11:** Development momentum index.

**Figure 12:** Satisfaction statistics of MICE tourism.

**Table 1:** Evaluation indexes for the development motivation mechanism of convention and exhibition tourism.

Factor	First-level evaluation index	Factor	Secondary evaluation index	Sort
*T*_1_	Economy	*S*_1_	Capital investment	3
		*S*_2_	Featured industry cluster	
		*S*_3_	International level	

*T*_2_	Resource	*S*_4_	Travel resources	1
		*S*_5_	Exhibition facilities	
		*S*_6_	Infrastructure	
		*S*_7_	Human resources	

*T*_3_	Location	*S*_8_	Political culture	2
		*S*_9_	Natural economy	
		*S*_10_	Regional market	

*T*_4_	Service	*S*_11_	Travel services	6
		*S*_12_	Expo services	

**Table 2:** Construction of evaluation indexes for motive mechanism of exhibition tourism development.

Factor	First-level evaluation index	Factor	Secondary evaluation index	Sort
*T*_5_	Policy	*S*_13_	Industrial policy	4
		*S*_14_	Exhibition system	
		*S*_15_	Government resources	

*T*_6_	Culture	*S*_16_	Citizen quality	7
		*S*_17_	The image of a city	
		*S*_18_	City safety	

*T*_7_	Technology	*S*_19_	Exhibition technology	5
		*S*_20_	Management technology	
		*S*_21_	Information technology	

**Table 3:** Judgment matrix of first-level index weight coefficient.

Power	*T*_1_	*T*_2_	*T*_3_	*T*_4_	*T*_5_	*T*_6_	*T*_7_	*W*
*T*_1_	1.97	1.85	2.68	2.12	1.11	2.08	2.86	0.1523
*T*_2_	1.55	2.85	1.98	1.82	2.96	2.98	1	0.2411
*T*_3_	1.66	1.33	2.2	1.11	2.1	2.05	1.36	0.1804
*T*_4_	2.79	2.39	2.58	2	1.42	1.33	2.59	0.0993
*T*_5_	2.89	1.76	2.5	1.17	2.33	1.8	1.73	0.1458
*T*_6_	2.6	1.66	2.02	1.01	1.53	1.6	2.05	0.0769
*T*_7_	1.32	2.75	1.71	1.54	1.23	2.97	2.82	0.1042

## Data Availability

The data used to support the findings of this study are available from the author upon request.
